The article "Berberine reduces temozolomide resistance by inducing autophagy via the ERK1/2 signaling pathway in glioblastoma" was retracted in 2024. Reasons: duplicated images; overlap with other authors' work; unreliable results or conclusions; concerns about the images.

# Berberine reduces temozolomide resistance by inducing autophagy via the ERK1/2 signaling pathway in glioblastoma

**DOI:** 10.1186/s12935-020-01693-y

**Published:** 2020-12-09

**Authors:** Huiling Qu, Xiaofu Song, Zhuyin Song, Xin Jiang, Xin Gao, Lijuan Bai, Jiao Wu, Li Na, Zhicheng Yao

**Affiliations:** 1 Department of Neurology, The People’s Hospital of Liaoning Province, 33 Wenyi Road, Shenhe District, Shenyang, 110016 Liaoning China; 2 Department of Laboratory Medicine, The People’s Hospital of Liaoning Province, Shenyang, Liaoning China

**Keywords:** Berberine, ERK1/2, GBM, Autophagy, Chemoresistance

## Abstract

**Background:**

The ability to treat glioblastoma (GBM) using the chemotherapeutic agent temozolomide (TMZ) has been hampered by the development of therapeutic resistance. In this study, we assessed the ability of the isoquinoline alkaloid berberine to alter GBM TMZ resistance using two different TMZ-resistant cell lines to mimic a physiologically relevant GBM experimental system.

**Methods:**

By treating these resistant cell lines with berberine followed by TMZ, we were able to assess the chemosensitivity of these cells and their parental strains, based on their performance in the MTT and colony formation assays, as well as on the degree of detectable apoptosis that was detected in the strains. Furthermore, we used Western blotting to assess autophagic responses in these cell lines, and we extended this work into a xenograft mouse model to assess the in vivo efficacy of berberine.

**Results:**

Through these experiments, our findings indicated that berberine enhanced autophagy and apoptosis in TMZ-resistant cells upon TMZ treatment in a manner that was linked with ERK1/2 signaling. Similarly, when used in vivo, berberine increased GBM sensitivity to TMZ through ERK1/2 signaling pathways.

**Conclusions:**

These findings demonstrate that berberine is an effective method of increasing the sensitization of GBM cells to TMZ treatment in a manner that is dependent upon the ERK1/2-mediated induction of autophagy, thus making berberine a potentially viable therapeutic agent for GBM treatment.

## Introduction

Of all the types of primary brain tumors affecting adults, glioblastoma (GBM) remains the deadliest [1, 2]. The standard approach for treatment involves the combination of surgical tumor excision and treatment with the chemotherapeutic agent temozolomide (TMZ), following the diagnosis of GBM [3–6]. However, even with such a treatment, the GBM prognosis remains poor, with a median survival time of less than 15 months in patients [7, 8]. TMZ resistance is extremely common among GBM patients undergoing therapeutic treatments, and such resistance serves as a barrier to the effective durable treatment of GBM [9–11]. Thus, it is important to study the mechanisms underlying TMZ resistance in an effort to develop novel sensitization strategies for clinical applications.

The article "Berberine reduces temozolomide resistance by inducing autophagy via the ERK1/2 signaling pathway in glioblastoma" was retracted in 2024. Reasons: duplicated images; overlap with other authors' work; unreliable results or conclusions; concerns about the images.

Autophagy is an evolutionarily conserved mechanism by which cells and organisms execute the ordered degradation and recycling of cells and cellular components [12, 13]. Autophagy has been linked with an array of physiologically important biological processes, with recent work suggesting a putative link between successful chemotherapeutic treatment and the induction of autophagy [14, 15]. Some studies have suggested that autophagy precedes the apoptotic cell death of GBM cells following TMZ administration, with observations indicating that compounds such as rapamycin (which can induce autophagy) may also be capable of enhancing the TMZ sensitivity of GBM cells, although not all studies have definitively supported this link [16–18]. Thus, the identification of novel strategies that are sufficient in altering autophagic responses for the treatment with chemotherapeutic compounds, such as TMZ, may be a viable strategy to reduce chemoresistance in GBM patients.

Berberine, which is an isoquinoline alkaloid derived from Huanglian (*Coptis chinensis*) and other traditional medicinal herbs, is among the most commonly utilized herbal medicines [19, 20]. A number of therapeutic properties have been attributed to berberine (in the context of cancer treatment), with such properties including the promotion of the induction of apoptosis in tumor cells and the further mediation of the growth arrest of tumor cells [21, 22].

In the current study, we aimed to test the ability of berberine to enhance TMZ sensitivity in GBM tumor cells, with a particular focus on the ERK1/2-mediated regulation of autophagy.

## Materials and methods

### Cell lines and reagents

U87 and U251 cells were obtained from The American Type Culture Collection (ATCC, USA) and were grown under standard conditions in DMEM media containing 10% fetal bovine serum (FBS; Gibco, Carlsbad, CA, USA) and 1% penicillin/streptomycin (Gibco). Berberine, TMZ, and 3-Methyladenine (3-MA) were obtained from Sigma-Aldrich (St. Louis, MO, USA). TMZ-resistant U87 and U251 cells were generated via an iterative treatment of the parental lines. The increasing TMZ concentration of 50–600 μM were used for selection of U87 and U251 cells, and the resistance cells were cultured in 300 μM TMZ. ERK1 plasmid was obtained from Addgene (#49328).

### Cell viability assay

The cell viability assay was performed as described by previous studies [23, 24]. Briefly, trypsin was used to harvest cells, which were then plated at 5 × 10^3^ per well in a 96-well plate. After 24 h, cells were treated with fresh media containing berberine and/or TMZ, as appropriate. These cells were then used in an MTT assay based on the provided manufacturer’s instructions, and the absorbance was measured at 490 nm as a correlate for cell viability.

The article "Berberine reduces temozolomide resistance by inducing autophagy via the ERK1/2 signaling pathway in glioblastoma" was retracted in 2024. Reasons: duplicated images; overlap with other authors' work; unreliable results or conclusions; concerns about the images.

### Colony formation assay

The colony formation assay was performed as described by previous studies [25, 26]. Cells were added to 6-well plates and treated by using the indicated compounds for 14 days under standard growth conditions, after which 0.1% crystal violet was used to stain for colonies that were then counted.

### Flow cytometry

A total of 500,000 cells were resuspended in 0.5 ml and stained for 15 min at room temperature by using 1.25 μl AnnexinV-FITC (Sigma). Stained cells were then centrifuged (1000 rpm, 5 min), resuspended in 0.5 ml cold binding buffer, and stained by using 10 μl propidium iodide (PI). Apoptosis was then analyzed via flow cytometry by using a quadrant-based gating strategy as follows: the viable cells were AnnexinV-/PI-, the cells in the early stages of apoptosis were Annexin V+/PI−, and the cells in the late stages of apoptosis were AnnexinV+/PI+. The overall rates of apoptosis were determined based on the total frequency of Annexin V+ cells.

### Western blot assay

Western blotting was performed as described by previous studies [27, 28]. Briefly, cellular protein was collected with the RIPA lysis buffer, and 10% SDS-PAGE gels were used to separate 50 μg protein per sample. The protein was then transferred to PVDF membranes that were blocked for 1 h at 37 °C with 5% skim milk. Blots were probed overnight at 4 °C by using 1:1000 primary antibodies against Beclin 1, LC3I/II, p62, cleaved caspase-3, Bax, Bcl-2, β-actin (Cell Signaling Technology, USA), ERK and p-ERK (Abcam, USA). Blots were then washed three times in TBST and probed for 1 h with HRP-conjugated goat anti-rabbit secondary antibody (Cell Signaling Technology, USA). Protein detection utilized a 1:1 combination reagent that was composed of peroxide and luminol (Millipore, USA).

### Immunoprecipitation

The indicated cells were harvested and suspended in 0.5 ml of cell lysis buffer supplemented with the protease inhibitor cocktail. After disruption of cells by sonication, cell lysates were collected by centrifugation at 12,000 ×g for 30 min. One mg of Bcl-2 antibody was mixed with protein G-agarose beads (Invitrogen) for 1 h at room temperature. The beads were washed thrice with TBS containing 0.02% Tween 20 (TBST), incubated with cell lysates on a rocker for overnight at 4 °C, and then washed thrice with TBS. Beads were then boiled in 2 × Laemmli buffer and subjected to Western blotting.

The article "Berberine reduces temozolomide resistance by inducing autophagy via the ERK1/2 signaling pathway in glioblastoma" was retracted in 2024. Reasons: duplicated images; overlap with other authors' work; unreliable results or conclusions; concerns about the images.

### Wound-healing assay

Wounds were generated via the use of a 200 µl pipette tip to scrape the GBM cultures. Healing was then observed via light microscopy over a 24-h time period, with the WimScratch Wimasis Image Analysis software being used to assess closure.

### Invasion assay

One hundred thousand cells were added to the upper chamber of a 24-well Multiwell insert (BD) that was coated with a 1:100 Matrigel solution. Culture media was then added to the lower chamber, and the plates were incubated for 72 h, after which cell migration into the lower chamber was assessed by fixing, Giemsa staining, and the counting of cells in the lower wells.

### Tumor xenograft model

The animal experiments were approved by the committee for animal experimentation of The People's Hospital of Liaoning Province and were performed in conjunction with the corresponding guidelines. BALB/c nude mice (6–8 weeks of age) received a flank injection of U87/TMZ-R cells. The mice were then intraperitoneally (i.p.) injected with TMZ (20 mg/kg), berberine (50 mg/kg), or the combined treatment of these drugs every other day for 19 days. Tumor volumes were determined based on the following formula: L × W^2^/2. After 19 days, the mice were euthanized, and tissue samples were collected for immunohistochemistry.

### Immunohistochemistry (IHC)

For immunohistochemistry, the cells were incubated in blocking solution and stained with primary antibody (1:100). Subsequent to the incubation with the suitable HRP-tethered antibodies (Bio-Rad, CA, USA) for 1 h, the signals were observed via the Diaminobenzidine Kit (Invitrogen, USA). The samples were then stained via hematoxylin and mounted with Acrymount. The specimens were observed through the use of an Olympus IX-81 microscope. The staining scores were assigned according to the percentage of positive tumor cells (0, 0%; 1, < 25%; 2, 25–50%; 3, 51–75%; and 4, > 75%) and staining intensity (0, none; 1, weakly stained; 2, moderately stained; and 3, strongly stained).

### Statistical analysis

Data are represented as the means ± standard deviation (SD), with all of the experiments conducted in triplicate. One-way analyses of variance (ANOVAs) were used for the between-group comparisons, and least significant difference tests were used for comparing the means of the two groups. The results with *p* < 0.05 were determined to be statistically significant.

## Results

### Berberine increases the TMZ sensitivity in TMZ-resistant GBM cells

To generate TMZ-resistant (TMZ-R) GBM cell lines, we intermittently treated the U87 and U251 cell lines with increasing TMZ doses (from 50 to 600 µM) over a 10-month time period. To assess TMZ resistance in these cells, we monitored the IC 50 values of their responses to TMZ treatment at three time points (24, 48, and 72 h), eventually generating the resultant U87/TMZ-R and U251/TMZ-R lines that were less sensitive to TMZ than their parental strains (Fig. 1a, b).

The article "Berberine reduces temozolomide resistance by inducing autophagy via the ERK1/2 signaling pathway in glioblastoma" was retracted in 2024. Reasons: duplicated images; overlap with other authors' work; unreliable results or conclusions; concerns about the images.

**Fig. 1:** Berberine resensitizes TMZ resistance cells to TMZ in GBM cells. **a** and **b** Parental and TMZ resistance cells were treated with increasing concentrations of TMZ for 24, 48 72 h. Cell viability was analyzed by MTT assay. **c** and **d** TMZ resistance cells were treated with TMZ with or without 10 μM berberine for 72 h. Cell viability was analyzed by MTT assay. **e** and **f** TMZ resistance cells were treated with 100 μM TMZ with or without 10 μM berberine for 72 h. Apoptosis was analyzed flow cytometry. **g** and **h** Parental and TMZ resistance cells were treated with 100 μM TMZ with or without 10 μM berberine as indicated for 24 h. Cleaved caspase 3 was analyzed by western blotting and normalized to β-actin. BBR: berberine. Results were presented as means ± SD from three independent experiments. **, *P* < 0.01

To determine whether berberine could alter the sensitivities of these cell lines to TMZ, the two TMZ-R lines were treated with berberine and then assessed via MTT and colony formation assays upon the TMZ treatment. To investigate the effect of berberine on TMZ resistance in GBM cells, we first determined the IC 50 of berberine in TMZ-R cells. Our data demonstrated that IC 50 values of berberine were more than 50 µM in the TMZ-R cells (Additional file 1: Figure S1A, B). Next, we used a lower concentration of berberine to show the combination effect. Berberine (10 µM) significantly increased the TMZ sensitivities of both U87/TMZ-R and U251/TMZ-R cells (Fig. 1c, d). Furthermore, we observed that the pretreatment with berberine resulted in higher rates of apoptosis in these TMZ-R cell lines upon TMZ treatment via the Annexin V/PI staining (Fig. 1e, f). Berberine-treated U87/TMZ-R and U251/TMZ-R cells also performed worse in response to the colony formation assays (Additional file 1: Figure S1C, D), and we confirmed the elevated rates of apoptosis in these cells by the use of western blotting (Fig. 1g, h). Taken together, these results support a role for berberine in sensitizing TMZ-R GBM cells to chemotherapeutic treatment.

### Berberine reduces the migration and invasion of TMZ-resistant GBM cells

With the use of wound-healing assays, we next tested whether a pretreatment with berberine would alter the migration and invasion potential of TMZ-R GBM cells. In cells that had been pretreated with berberine, we observed a significant reduction in both the U87/TMZ-R and U251/TMZ-R cell lines at 24 h following wound generation (Fig. 2a–d), thus indicating a berberine-dependent disruption of the migratory potential in these cells.

The article "Berberine reduces temozolomide resistance by inducing autophagy via the ERK1/2 signaling pathway in glioblastoma" was retracted in 2024. Reasons: duplicated images; overlap with other authors' work; unreliable results or conclusions; concerns about the images.

**Fig. 2:** Berberine inhibits migration and invasion in TMZ resistance GBM cells. **a** and **b** TMZ resistance U87 cells were treated with 100 μM TMZ with or without 10 μM berberine for 24 h. The migration (wound healing) ability was analyzed as indicated. **c** and **d** TMZ resistance U251 cells were treated with 100 μM TMZ with or without 10 μM berberine for 24 h. The migration (wound healing) ability was analyzed as indicated. **e** TMZ resistance U87 cells were treated with 100 μM TMZ with or without 10 μM berberine for 24 h. The invasion ability was analyzed as indicated. **f** TMZ resistance U251 cells were treated with 100 μM TMZ with or without 10 μM berberine for 24 h. The invasion ability was analyzed as indicated. BBR: berberine. Results were presented as means ± SD from three independent experiments. *, *P* < 0.05

To further confirm and extend these findings, we used both the parental and TMZ-R lines of the U87 and U251 cells in a chamber-based invasion assay. Following the pretreatment with berberine, we counted the number of cells that were able to migrate through the Matrigel layers into the lower chambers in each treatment condition (Fig. 2e, f, Additional file 1: Figure S2A, B). Interestingly, the pretreatment with berberine disrupted this invasive ability in both the parental and resistant cells. Therefore, berberine may have anti-invasive effects that affect TMZ sensitivity.

### Berberine promotes TMZ-induced autophagy in GBM cells

Previous studies have demonstrated that autophagy is involved in TMZ resistance in GBM cells [29]. Our findings indicated significantly reduced autophagy in the U87/TMZ-R and U251/TMZ-R cells relative to their parental cell lines (Fig. 3a, b), which is consistent with a previous study that described a role for autophagy in promoting chemosensitivity. This phenomenon may explain the enhanced TMZ resistance that was observed in this cell line. TMZ resistance in previously untreated GBM patients is mediated predominantly by the *O*^6^-methylguanine-DNA methyltransferase (MGMT) protein [30]. Our findings indicated that MGMT has nothing to do with berberine-induced TMZ sensitization in TMZ-R cells (Additional file 1: Figure S3A, B).

**Fig. 3:** Berberine promotes TMZ-induced autophagy in TMZ-R cells. **a** and **b** The indicated protein level was analyzed by western blotting in parental and TMZ resistance cells. LC3 II was normalized to LC3 I. **c** TMZ-R U87 cells were transfected with GFP-LC3 plasmid, followed by treatment with 100 μM TMZ with or without 10 μM berberine for 24 h. The numbers of GFP-LC3 puncta were quantified with confocal microscopy. **d** TMZ-R U251 cells were transfected with GFP-LC3 plasmid, followed by treatment with 100 μM TMZ with or without 10 μM berberine for 24 h. The numbers of GFP-LC3 puncta were quantified with confocal microscopy. **e** and **f** TMZ resistance cells were treated with 100 μM TMZ with or without 10 μM berberine as indicated for 24 h. Indicated proteins level were analyzed by western blotting. LC3 II was normalized to LC3 I. **g** and **h** TMZ resistance cells were treated with 100 μM TMZ and 10 μM berberine as indicated time points. Indicated proteins level were analyzed by western blotting. LC3 II was normalized to LC3 I. BBR: berberine. Results were presented as means ± SD from three independent experiments. *, *P* < 0.05

Therefore, we assessed whether the pretreatment with berberine altered rates of autophagy in U87/TMZ-R cells by using a GFP-LC3 construct, in order to visualize the rates of autophagy via immunofluorescence microscopy. We observed increased rates of GFP+ vesicles in these cells upon TMZ treatment in cells with a pretreatment with berberine (Fig. 3c, d, Additional file 1: Figure S3C, D). We further performed western blotting to assess LC3-II, p62, and Beclin-1 levels as protein readouts for the rates of cellular autophagy, with all 3 of these levels being observed to be elevated in the TMZ-treated TMZ-R cells that were first pretreated with berberine (Fig. 3e, f). In addition, the combination treatment induced autophagy in a time-dependent manner (Fig. 3g, h). These findings suggest that berberine induces autophagy in TMZ-R cell lines, thus potentially sensitizing them to subsequent cell death.

The article "Berberine reduces temozolomide resistance by inducing autophagy via the ERK1/2 signaling pathway in glioblastoma" was retracted in 2024. Reasons: duplicated images; overlap with other authors' work; unreliable results or conclusions; concerns about the images.

### Berberine promotes TMZ sensitivity via the induction of autophagy

To further investigate the role of autophagy as a means of sensitizing cells to TMZ in this model system, we assessed the relationship between autophagy and apoptosis in berberine-treated U87/TMZ-R cells. By treating cells with 3-MA, which inhibits autophagy, we were able to eliminate the observed berberine-dependent disruption of cell viability and colony formation in these TMZ-R cells (Fig. 4a, b, Additional file 1: Figure S4A, B).

**Fig. 4:** Autophagy induction is required for berberine-induced TMZ resensitization in TMZ-R cells. **a** and **b** TMZ resistance cells were treated with increasing concentrations of TMZ with or without berberine and 1 mM 3-MA for 72 h. Cell viability was analyzed by MTT assay. **c** and **d** TMZ resistance cells pretreated with 1 mM 3-MA were treated with 100 μM TMZ with or without 10 μM berberine for 24 h. Apoptosis was analyzed flow cytometry. **e** and **f** TMZ resistance cells pretreated with 1 mM 3-MA were treated with 100 μM TMZ with or without 10 μM berberine for 24 h. Indicated proteins level were analyzed by western blotting. LC3 II was normalized to LC3 I. BBR: berberine. Results were presented as means ± SD from three independent experiments. *, *P* < 0.05

This result was further demonstrated by the fact that 3-MA decreased the combination treatment of TMZ and berberine-induced apoptosis in U87/TMZ-R and U251/TMZ-R cells (Fig. 4c, d). In addition, the combination treatment-induced apoptosis was attenuated by bafilomycin A1 in U87/TMZ-R and U251/TMZ-R cells (Additional file 1: Figure S4C, D). The treatment of U87/TMZ-R cells with 3-MA also reduced both caspase-3 activation and LC3-I-to-LC3-II conversion in these cells following a TMZ and berberine cotreatment (Fig. 4e, f). This result supports the idea of a direct autophagy-dependent role for berberine in its ability to enhance the apoptotic cell death of TMZ-R GBM cells.

### Berberine induces autophagy via the ERK1/2 signaling pathway

Previous studies have demonstrated that the berberine treatment of GBM cells can downregulate the activation of EGFR/MEK/ERK1/2 signaling, thus suggesting a potential role for ERK1/2 signaling in the present autophagy-dependent system [31, 32]. Therefore, we analyzed the MAPK signaling pathways in the parental and TMZ resistance cells. Our findings demonstrated that the ERK1/2 signaling pathway becomes significantly activated in the TMZ-R cell lines (Fig. 5a, b).

**Fig. 5:** Berberine induces autophagy via ERK signaling inhibition. **a** and **b** Total and phosphorylation ERK was analyzed by western blotting in parental and TMZ resistance cells. **c** and **d** TMZ-R U87 and U251 cells were transfected with GFP-LC3 with or without ERK1 plasmid, followed by treatment with 100 μM TMZ with 10 μM berberine for 24 h. The numbers of GFP-LC3 puncta were quantified with confocal microscopy. **e** and **f** TMZ-R U87 and U251 cells were transfected with ERK1 plasmid, followed by treatment with 100 μM TMZ with 10 μM berberine for 24 h. Indicated proteins level were analyzed by western blotting. LC3 II was normalized to LC3 I. **g** IP experiment was performed with antibody against Bcl-2 in berberine-treated TMZ-R cells. Then the Beclin1 was analyzed by western blotting. BBR: berberine. Results were presented as means ± SD from three independent experiments. *, *P* < 0.05

The overexpression of ERK1 in U87/TMZ-R cells reduced the ability of berberine to induce autophagy in these cells (Fig. 5c, d). Western blotting further confirmed this ERK1/2-dependent suppression of berberine-induced autophagy (Fig. 5e, f). Moreover, we performed IP experiment to detect the interaction of Beclin1 and Bcl-2 upon berberine treatment in TMZ-R cells. The IP results revealed that berberine decreased the interaction of Bcl-2 and Beclin1 (Fig. 5g). Our results demonstrated that ERK1/2 signaling is essential for TMZ-mediated autophagy induction in this GBM cell line.

The article "Berberine reduces temozolomide resistance by inducing autophagy via the ERK1/2 signaling pathway in glioblastoma" was retracted in 2024. Reasons: duplicated images; overlap with other authors' work; unreliable results or conclusions; concerns about the images.

### Berberine increases GBM TMZ sensitivity in vivo

To extend these findings in vivo, we employed the U87/TMZ-R cells in a mouse xenograft model. After a subcutaneous flank implant with the tumor cells, mice were administered TMZ, berberine, and the combination of these drugs. We observed that berberine treatment reduced tumor weights and tumor growth rates in mice that were implanted with U87/TMZ-R cells, relative to the TMZ-only controls (Fig. 6a, b). We further observed that the treatment with berberine was associated with increased tumor expression levels of LC3II, Bax, and active caspase-3, as well as decreased phospho-ERK1/2 and Bcl-2 levels (Fig. 6c). The upregulation of LC3B and active caspase 3 expression levels was confirmed via immunohistochemical tests (Fig. 6d, e, Additional file 1: Figure S6A, B). These results support our in vitro results, thus suggesting that berberine can promote an increase in TMZ sensitivity via the ERK1/2- and autophagy-dependent pathways.

**Fig. 6:** Berberine resensitizes TMZ to TMZ-R tumors in vivo. **a** Nude mice were injected s.c. with 4 × 10^6 ^TMZ-R cells. After 1 week, mice were treated with TMZ, berberine or their combination. Tumor volume was calculated and plotted with p values, n = 6 in each group. **b** Tumor weight at the end of the experiment. **c** The indicated proteins in randomly selected tumors were analyzed by Western blotting. LC3 II was normalized to LC3 I. **d** Paraffin-embedded sections of TMZ-R tumor tissues from mice treated were analyzed by active caspase 3 staining. **e** Paraffin-embedded sections of TMZ-R tumor tissues from mice treated were analyzed by LC3B staining. BBR: berberine. Results were presented as means ± SD from three independent experiments. *, *P* < 0.05

## Discussion

Globally, GBM is the deadliest type of brain tumor; even with aggressive surgical and chemotherapeutic treatments, the median survival time following diagnosis is still < 15 months [33, 34]. The treatment with TMZ remains the standard approach for treating GBM [35, 36]. However, the relatively quick development of chemoresistance to this compound limits the efficacy of this therapeutic strategy [36]. Currently, a number of different and distinct mechanisms of TMZ resistance have been identified by researchers, including mechanisms that are dependent upon DNA *O*^6^-methylguanine methyltransferase (MGMT), DNA mismatch repair (MMR), base excision repair (BER), and the ATP-binding cassette (ABC) protein family [37–40]. Given these diverse mechanisms and the key role of TMZ in treating GBM, it is clear that more research needs to be performed to determine how TMZ resistance develops and what strategies are effective in increasing the sensitivity of TMZ-R cell lines to chemotherapeutic treatments.

The article "Berberine reduces temozolomide resistance by inducing autophagy via the ERK1/2 signaling pathway in glioblastoma" was retracted in 2024. Reasons: duplicated images; overlap with other authors' work; unreliable results or conclusions; concerns about the images.

In the present study, we utilized TMZ-R GBM cell lines in order to demonstrate the ability of berberine to restore TMZ sensitivity to these cells, as well as the demonstration of the further berberine-dependent suppression of cellular migration and invasive potential. These results seem to be at least partially linked to a berberine-dependent induction of autophagy and apoptosis, although the exact underlying molecular mechanisms remain to be fully determined.

Different studies have highlighted roles for autophagy in promoting both the survival and apoptotic death of GBM cells, thus suggesting that the specific treatment context determines the therapeutic value of this complex physiological process [41, 42]. Even so, previous data support a link between reduced autophagy and the resistance to chemotherapy in GBM cells [9]. Consistent with such findings, we observed significant reductions in baseline autophagy in TMZ-R cells, relative to the parental strain. Berberine was able to enhance TMZ sensitivity in this resistant cell line, and this effect was ablated following the treatment with the autophagy inhibitor 3-MA, thus suggesting that berberine acts (at least partially) via autophagy induction.

More studies are needed to fully elucidate how berberine may modulate autophagy in TMZ-R GBM cells. Previous studies have indicated that ERK1/2/Bcl-2/Beclin-1 signaling is linked to autophagy induction and that berberine can suppress ERK1/2 signaling in glioma cells, in order to suppress tumor growth [43, 44]. Consistent with these previous studies, we observed ERK1/2-dependent alterations in autophagy upon berberine treatment in U87/TMZ-R cells, thus suggesting that berberine can induce autophagy (at least partially) by altering ERK1/2 signaling in vitro and in vivo. Previous studies have shown that berberine regulating Wnt/β-catenin, JAK-STAT, mTOR pathway in cancer cells [45]. Berberine may induced autophagy in human liver carcinoma cell lines via Beclin-1 activation [46]. Several researchers pointed out to a correlation between berberine treatment and expression of non-coding RNAs, either lncRNAs or microRNAs [47]. It was shown that berberine suppresses interleukin 6 (IL-6), a factor required for cell growth in multiple myeloma cells (U266), through negative regulation of the STAT3, and this induces inhibition of miR-21 expression [48]. Recent studies have also highlighted a role for autophagy as a means of inducing apoptotic cell death in GBM cells, with ERK1/2/Bcl-2/Beclin-1 signaling being linked to such autophagy induction [44, 49, 50]. ERK1/2 can promote the activation of Bcl-2 transcription, thereby inhibiting the induction of autophagy via the dissociation of the Bcl-2/Beclin-1 complex [51].

The article "Berberine reduces temozolomide resistance by inducing autophagy via the ERK1/2 signaling pathway in glioblastoma" was retracted in 2024. Reasons: duplicated images; overlap with other authors' work; unreliable results or conclusions; concerns about the images.

In conclusion, our present study highlights a potential role for berberine as a method of increasing the chemosensitivity of GBM tumors. We demonstrated that the pretreatment with berberine was sufficient to enhance GBM TMZ-sensitivity in both cell cultures and murine xenograft systems, with a clear role for berberine in the ERK1/2-dependent induction of autophagy and in the apoptosis of these TMZ-R GBM cells. This result suggests that the combination of berberine with TMZ may be a viable method of enhancing patient responses to therapy.

## Supplementary Information

**Additional file 1: Figure S1.** **(A)** U87 TMZ-R cells were treated with increasing concentration of berberine for 72 hours. Cell viability was analyzed by MTT assay. **(B)** U251 TMZ-R cells were treated with increasing concentration of berberine for 72 hours. Cell viability was analyzed by MTT assay. **(C)** and **(D)** TMZ resistance cells were treated with 100 μM TMZ with or without 10 μM berberine for 24 hrs. Colony formation assays were repeated at least three times. Results were presented as means ± SD from three independent experiments. **, *P* < 0.01.** Figure S2.** **(A)** TMZ resistance U87 cells were treated with 100 μM TMZ with or without 10 μM berberine for 24 hrs. The invasion ability was analyzed as indicated. **(B)** TMZ resistance U251 cells were treated with 100 μM TMZ with or without 10 μM berberine for 24 hrs. The invasion ability was analyzed as indicated. BBR: berberine. **Figure S3.** **(A)** Western blotting of MGMT in U87 and U87/TMZ-R cells.** (B)** U87/TMZ-R cells were treated with 10 μM berberine at indicated time points. MGMT was analyzed by western blotting.** (C)** and **(D)** TMZ-R U87 cells were transfected with GFP-LC3 plasmid, followed by treatment with 100 μM TMZ with or without 10 μM berberine for 24 hrs. The numbers of GFP-LC3 puncta were quantified with confocal microscopy. **Figure S4.** **(A)** and **(B)** TMZ resistance cells pretreated with 1 mM 3-MA were treated with 100 μM TMZ with or without 10 μM berberine for 24 hrs. Colony formation assays were repeated at least three times.** (C)** and **(D)** TMZ resistance cells pretreated with bafilomycin A1 (10 nM) were treated with 100 μM TMZ with or without 10 μM berberine for 24 hrs. Apoptosis was analyzed flow cytometry. **Figure S5.** **(A)** Paraffin-embedded sections of TMZ-R tumor tissues from mice treated were analyzed by active caspase 3 staining. Scale bar: 25μm. BBR: berberine.** (B)** Paraffin-embedded sections of TMZ-R tumor tissues from mice treated were analyzed by LC3B staining. Scale bar: 25μm. BBR: berberine.

The article "Berberine reduces temozolomide resistance by inducing autophagy via the ERK1/2 signaling pathway in glioblastoma" was retracted in 2024. Reasons: duplicated images; overlap with other authors' work; unreliable results or conclusions; concerns about the images.

## Data Availability

The data supporting the findings of this study are available from the corresponding author upon request.

## Abbreviations

3-MA: 3-Methyladenine
ABC: ATP-binding cassette
ATCC: American Type Culture Collection
BER: Base excision repair
FBS: Fetal bovine serum
GBM: Glioblastoma
IHC: Immunohistochemistry
MGMT: *O*^6^-methylguanine methyltransferase
MMR: Mismatch repair
SD: Standard deviation
TMZ: Temozolomide

## References

[1] Davis ME (2016). Glioblastoma: overview of disease and treatment. Clin J Oncol Nurs.

[2] Lim M, Xia Y, Bettegowda C, Weller M (2018). Current state of immunotherapy for glioblastoma. Nat Rev Clin Oncol.

[3] Paolillo M, Boselli C, Schinelli S (2018). Glioblastoma under Siege: an overview of current therapeutic strategies. Brain Sci.

[4] Noroxe DS, Poulsen HS, Lassen U (2016). Hallmarks of glioblastoma: a systematic review. ESMO Open.

[5] Tseng WL, Hsu HH, Chen Y, Tseng SH (2017). Tumor recurrence in a glioblastoma patient after discontinuation of prolonged temozolomide treatment. Asian J Neurosurg.

[6] Mallick S, Gandhi AK, Rath GK (2015). Therapeutic approach beyond conventional temozolomide for newly diagnosed glioblastoma: review of the present evidence and future direction. Indian J Med Paediatr Oncol.

[7] Delgado-Lopez PD, Corrales-Garcia EM (2016). Survival in glioblastoma: a review on the impact of treatment modalities. Clin Transl Oncol.

[8] Shergalis A, Bankhead A, Luesakul U, Muangsin N, Neamati N (2018). Current challenges and opportunities in treating glioblastoma. Pharmacol Rev.

[9] Lee SY (2016). Temozolomide resistance in glioblastoma multiforme. Genes Dis.

[10] Goellner EM, Grimme B, Brown AR, Lin YC, Wang XH, Sugrue KF, Mitchell L, Trivedi RN, Tang JB, Sobol RW (2011). Overcoming temozolomide resistance in glioblastoma via dual inhibition of NAD+ biosynthesis and base excision repair. Cancer Res.

[11] Chen X, Zhang M, Gan H, Wang H, Lee JH, Fang D, Kitange GJ, He L, Hu Z, Parney IF, Meyer FB, Giannini C, Sarkaria JN, Zhang Z (2018). A novel enhancer regulates MGMT expression and promotes temozolomide resistance in glioblastoma. Nat Commun.

[12] Glick D, Barth S, Macleod KF (2010). Autophagy: cellular and molecular mechanisms. J Pathol.

The article "Berberine reduces temozolomide resistance by inducing autophagy via the ERK1/2 signaling pathway in glioblastoma" was retracted in 2024. Reasons: duplicated images; overlap with other authors' work; unreliable results or conclusions; concerns about the images.

[13] Ravikumar B, Sarkar S, Davies JE, Futter M, Garcia-Arencibia M, Green-Thompson ZW, Jimenez-Sanchez M, Korolchuk VI, Lichtenberg M, Luo S, Massey DC, Menzies FM, Moreau K, Narayanan U, Renna M, Siddiqi FH, Underwood BR, Winslow AR, Rubinsztein DC (2010). Regulation of mammalian autophagy in physiology and pathophysiology. Physiol Rev.

[14] Sui X, Chen R, Wang Z, Huang Z, Kong N, Zhang M, Han W, Lou F, Yang J, Zhang Q, Wang X, He C, Pan H (2013). Autophagy and chemotherapy resistance: a promising therapeutic target for cancer treatment. Cell Death Dis.

[15] Shimizu S, Nakao K, Minato N, Uemoto S (2015). Autophagic cell death and cancer chemotherapeutics. Innovative medicine.

[16] Moghadam AR, da Silva Rosa SC, Samiei E, Alizadeh J, Field J, Kawalec P, Thliveris J, Akbari M, Ghavami S, Gordon JW (2018). Autophagy modulates temozolomide-induced cell death in alveolar Rhabdomyosarcoma cells. Cell Death Discov.

[17] Kanzawa T, Germano IM, Komata T, Ito H, Kondo Y, Kondo S (2004). Role of autophagy in temozolomide-induced cytotoxicity for malignant glioma cells. Cell Death Differ.

[18] Li H, Chen L, Li JJ, Zhou Q, Huang A, Liu WW, Wang K, Gao L, Qi ST, Lu YT (2018). miR-519a enhances chemosensitivity and promotes autophagy in glioblastoma by targeting STAT3/Bcl2 signaling pathway. J Hematol Oncol.

[19] Neag MA, Mocan A, Echeverria J, Pop RM, Bocsan CI, Crisan G, Buzoianu AD (2018). Berberine: botanical occurrence, traditional uses, extraction methods, and relevance in cardiovascular, metabolic, hepatic, and renal disorders. Front Pharmacol.

[20] Hesari A, Ghasemi F, Cicero AFG, Mohajeri M, Rezaei O, Hayat SMG, Sahebkar A (2018). Berberine: aa potential adjunct for the treatment of gastrointestinal cancers?. J Cell Biochem.

[21] Jin Y, Khadka DB, Cho WJ (2016). Pharmacological effects of berberine and its derivatives: a patent update. Expert Opin Ther Pat.

[22] Ortiz LM, Lombardi P, Tillhon M, Scovassi AI (2014). Berberine, an epiphany against cancer. Molecules.

[23] Tong J, Zheng X, Tan X, Fletcher R, Nikolovska-Coleska Z, Yu J, Zhang L (2018). Mcl-1 phosphorylation without degradation mediates sensitivity to HDAC inhibitors by liberating BH3-only proteins. Cancer Res.

[24] Tong J, Wang P, Tan S, Chen D, Nikolovska-Coleska Z, Zou F, Yu J, Zhang L (2017). Mcl-1 degradation is required for targeted therapeutics to eradicate colon cancer cells. Cancer Res.

[25] Tong J, Tan S, Nikolovska-Coleska Z, Yu J, Zou F, Zhang L (2017). FBW7-ddependent Mcl-1 degradation mediates the anticancer effect of Hsp90 inhibitors. Mol Cancer Ther.

[26] Tong J, Tan S, Zou F, Yu J, Zhang L (2017). FBW7 mutations mediate resistance of colorectal cancer to targeted therapies by blocking Mcl-1 degradation. Oncogene.

The article "Berberine reduces temozolomide resistance by inducing autophagy via the ERK1/2 signaling pathway in glioblastoma" was retracted in 2024. Reasons: duplicated images; overlap with other authors' work; unreliable results or conclusions; concerns about the images.

[27] He K, Chen D, Ruan H, Li X, Tong J, Xu X, Zhang L, Yu J (2016). BRAFV600E-dependent Mcl-1 stabilization leads to everolimus resistance in colon cancer cells. Oncotarget.

[28] Chen D, Tong J, Yang L, Wei L, Stolz DB, Yu J, Zhang J, Zhang L (2018). PUMA amplifies necroptosis signaling by activating cytosolic DNA sensors. Proc Natl Acad Sci U S A.

[29] Yan Y, Xu Z, Dai S, Qian L, Sun L, Gong Z (2016). Targeting autophagy to sensitive glioma to temozolomide treatment. J Exp Clin Cancer Res.

[30] Kitange GJ, Carlson BL, Schroeder MA, Grogan PT, Lamont JD, Decker PA, Wu W, James CD, Sarkaria JN (2009). Induction of MGMT expression is associated with temozolomide resistance in glioblastoma xenografts. Neuro Oncol.

[31] Liu Q, Xu X, Zhao M, Wei Z, Li X, Zhang X, Liu Z, Gong Y, Shao C (2015). Berberine induces senescence of human glioblastoma cells by downregulating the EGFR-MEK-ERK signaling pathway. Mol Cancer Ther.

[32] Liu J, Zhao X, Pei D, Sun G, Li Y, Zhu C, Qiang C, Sun J, Shi J, Dong Y, Gou J, Wang S, Li A (2018). The promotion function of Berberine for osteogenic differentiation of human periodontal ligament stem cells via ERK-FOS pathway mediated by EGFR. Sci Rep.

[33] Zhang Y, Dube C, Gibert M, Cruickshanks N, Wang B, Coughlan M, Yang Y, Setiady I, Deveau C, Saoud K, Grello C, Oxford M, Yuan F, Abounader R (2018). The p53 Pathway in Glioblastoma. Cancers (Basel).

[34] Lee E, Yong RL, Paddison P, Zhu J (2018). Comparison of glioblastoma (GBM) molecular classification methods. Semin Cancer Biol.

[35] von Neubeck C, Seidlitz A, Kitzler HH, Beuthien-Baumann B, Krause M (2015). Glioblastoma multiforme: emerging treatments and stratification markers beyond new drugs. Br J Radiol.

[36] Munoz JL, Rodriguez-Cruz V, Walker ND, Greco SJ, Rameshwar P (2015). Temozolomide resistance and tumor recurrence: halting the Hedgehog. Cancer Cell Microenviron.

[37] Chen Z, Wei X, Shen L, Zhu H, Zheng X (2018). 20(S)-ginsenoside-Rg3 reverses temozolomide resistance and restrains epithelial-mesenchymal transition progression in glioblastoma. Cancer Sci.

[38] Perazzoli G, Prados J, Ortiz R, Caba O, Cabeza L, Berdasco M, Gonzalez B, Melguizo C (2015). Temozolomide resistance in glioblastoma cell lines: implication of MGMT, MMR, P-glycoprotein and CD133 expression. PLoS ONE.

[39] Zhang J, Stevens MF, Bradshaw TD (2012). Temozolomide: mechanisms of action, repair and resistance. Curr Mol Pharmacol.

[40] Pessina S, Cantini G, Kapetis D, Cazzato E, Di Ianni N, Finocchiaro G, Pellegatta S (2016). The multidrug-resistance transporter Abcc3 protects NK cells from chemotherapy in a murine model of malignant glioma. Oncoimmunology.

The article "Berberine reduces temozolomide resistance by inducing autophagy via the ERK1/2 signaling pathway in glioblastoma" was retracted in 2024. Reasons: duplicated images; overlap with other authors' work; unreliable results or conclusions; concerns about the images.

[41] Noonan J, Zarrer J, Murphy BM (2016). Targeting autophagy in glioblastoma. Crit Rev Oncog.

[42] Taylor MA, Das BC, Ray SK (2018). Targeting autophagy for combating chemoresistance and radioresistance in glioblastoma. Apoptosis.

[43] Regulation of the Autophagic Bcl-2/Beclin 1 InteractionMarquez RT and Xu L (2012). Bcl-2: Beclin 1 complex: multiple, mechanisms regulating autophagy/apoptosis toggle switch. Am J Cancer Res.

[44] Decuypere JP, Parys JB, Bultynck G (2012). Regulation of the autophagic bcl-2/beclin 1 interaction. Cells.

[45] Wang Y, Liu Y, Du X, Ma H, Yao J (2020). The anti-cancer mechanisms of berberine: a review. Cancer Manag Res.

[46] Deng Y, Xu J, Zhang X, Yang J, Zhang D, Huang J, Lv P, Shen W, Yang Y (2014). Berberine attenuates autophagy in adipocytes by targeting BECN1. Autophagy.

[47] Chang W (2017). Non-coding RNAs and Berberine: a new mechanism of its anti-diabetic activities. Eur J Pharmacol.

[48] Hu HY, Li KP, Wang XJ, Liu Y, Lu ZG, Dong RH, Guo HB, Zhang MX (2013). Set9, NF-kappaB, and microRNA-21 mediate berberine-induced apoptosis of human multiple myeloma cells. Acta Pharmacol Sin.

[49] He C, Zhu H, Li H, Zou MH, Xie Z (2013). Dissociation of Bcl-2-Beclin1 complex by activated AMPK enhances cardiac autophagy and protects against cardiomyocyte apoptosis in diabetes. Diabetes.

[50] Pattingre S, Tassa A, Qu X, Garuti R, Liang XH, Mizushima N, Packer M, Schneider MD, Levine B (2005). Bcl-2 antiapoptotic proteins inhibit Beclin 1-dependent autophagy. Cell.

[51] Kang R, Zeh HJ, Lotze MT, Tang D (2011). The Beclin 1 network regulates autophagy and apoptosis. Cell Death Differ.

